# *Uncaria tomentosa* for Reducing Side Effects Caused by Chemotherapy in CRC Patients: Clinical Trial

**DOI:** 10.1155/2012/892182

**Published:** 2011-08-21

**Authors:** I. L. G. Farias, M. C. S. Araújo, J. G. Farias, L. V. Rossato, L. I. Elsenbach, S. L. Dalmora, N. M. P. Flores, M. Durigon, I. B. M. Cruz, V. M. Morsch, M. R. C. Schetinger

**Affiliations:** ^1^Departamento de Química, Universidade Federal de Santa Maria, 97105-900 Santa Maria, RS, Brazil; ^2^Hospital Universitário de Santa Maria, Universidade Federal de Santa Maria, 97105-900 Santa Maria, RS, Brazil; ^3^Departamento de Biologia, Universidade Federal de Santa Maria, 97105-900 Santa Maria, RS, Brazil; ^4^Departamento de Farmácia Industrial, Universidade Federal de Santa Maria, 97105-900 Santa Maria, RS, Brazil; ^5^Departamento de Morfologia, Universidade Federal de Santa Maria, 97105-900 Santa Maria, RS, Brazil

## Abstract

To evaluate the effectiveness of *Uncaria tomentosa* in minimizing the side effects of chemotherapy and improving the antioxidant status of colorectal cancer (CRC) patients, a randomized clinical trial was conducted. Patients (43) undergoing adjuvant/palliative chemotherapy with 5-Fluorouracil/leucovorin + oxaliplatin (FOLFOX4) were split into two groups: the UT group received chemotherapy plus 300 mg of *Uncaria tomentosa* daily and the C group received only FOLFOX4 and served as a control. Blood samples were collected before each of the 6 cycles of chemotherapy, and hemograms, oxidative stress, enzymes antioxidants, immunologic parameters, and adverse events were analyzed. The use of 300 mg of *Uncaria tomentosa* daily during 6 cycles of FOLFOX4 did not change the analyzed parameters, and no toxic effects were observed.

## 1. Introduction

After histological diagnosis of colorectal cancer, the treatment of advanced stages of cancer involves adjuvant or palliative chemotherapy.One common treatment plan includes the application of 5-fluoruracil (5FU)/leucovorin and oxaliplatin (FOLFOX4) [1]. However, side effects from this treatment include severe neutropenia (grade 3 or 4 according to Common Toxicity Criteria of the National Cancer Institute) in 41.1% of patients [1]. Besides the cytotoxic effect of the chemotherapy, the cause of the neutropenia may be related to oxidative stress, because high H_2_O_2_ levels may negatively influence the proliferation and differentiation of myeloid precursors [2]. There is a well-documented relationship between oxidative stress and colorectal cancer. Oxidative stress may result in both DNA damage [3] and the expansion of neoplastic cells, because tumoral metabolic adaptations generate high level of reactive oxygen species (ROS) [4]. Additionally, chemotherapeutic cancer treatments increase oxidative stress levels [5], resulting in high levels of reactive oxygen species (ROS) and damage to the lipids of the cytoplasmic membrane, cellular proteins, and DNA [2].

The immune status of patients, particularly CD8^+^ and CD4^+^ T cells (T_regs_) levels, shows a correlation with survival. The CD4^+^/CD8^+^ ratio of the tumor infiltrating lymphocytes is significantly associated with colorectal cancer prognosis [6]. Treatment with 5FU increases IFN-*γ* production through the action of tumor-specific CD8^+^ T cells that infiltrate the tumor, and it promotes T cell-dependent antitumor responses *in vivo* [7]. Again, there is an interaction between the immune response and oxidative stress. Exposure to reactive oxygen species (ROS) produced by activated granulocytes and macrophages in the context of malignant disorders causes dysfunction of T-cells and NK cells [8]. High levels of superoxide dismutase (SOD—an antioxidant enzyme) contribute to tumor cell resistance and therapy insensitivity and are correlated with poor outcome [9].

For these reasons, it is important to search for complementary treatments, including phytotherapic plants, that minimize the neutropenia associated with colon cancer chemotherapy. *Uncaria tomentosa *(*Ut*, Cat's claw) has antioxidant properties [10] and can stimulate DNA repair [11] and myelopoiesis [12]. Eberlin et al. [12] showed that *Ut* extract promotes proliferation of myeloid precursors through the increase in serum colony stimulating growth factors (CSFs). Other preclinical experiments have demonstrated the positive effect of aqueous *Ut* extract on leukocyte counts over a period of eight weeks in healthy animals [13] and after ten days of doxorubicin-induced neutropenia [14]. Given these characteristics, *Ut* could minimize the undesirable effects of chemotherapy and might improve the balance between stress and antioxidants in cancer patients. This clinical study aimed to evaluate the effect of coadjuvant treatment with *Ut* compared with conventional chemotherapy for colorectal cancer. The investigation evaluated the effect of *Ut* on oxidative stress and its consequences in relation to neutropenia, other hematological parameters, immune system, safety, and side effects.

## 2. Methods

### 2.1. Design and Patients

We performed a randomized interventional study of colorectal cancer patients who were submitted to chemotherapy treatment. 

The study was carried out with 43 patients (26 female, 17 male) who had undergone complete resection of their colorectal cancer, which was of histologically scored as stage IIB, III, or IV, and who were going to begin adjuvant/palliative chemotherapy with FOLFOX4 at the *Hospital Universitário de Santa Maria*, Brazil. 

Patients were randomly grouped into two groups, according to the date of treatment start as follows: the first patient who agreed participating in the study was included into UT group, the second into the C group, and successively until the end. The UT group was treated with FOLFOX4 plus *Ut*, and the control group (C) received only FOLFOX4. Patients remained on study during 6 chemotherapies cycles, of 15 days each. The doses of medication in UT group were as follows: Oxaliplatin, 85 mg/m² on day1; 5FU, 1 g/m² on days 1 and 2; Leucovorin, 200 mg/m² on days 1 and 2; and *Ut* (Unha de Gato Herbarium), 3 tablets daily from day 3 to day 15. The dose of *Ut *is similar to that used in previous study, using 250–350 mg C-MED-100, an aqueous extracts of *Ut* [11]. No changes in food intake pattern had occurred during the supplementation.

The calculation for estimating the sample size required for a randomized clinical trial was according to Greenberg et al. [15], with constant level of significance (*α*) of 5%, and statistical power of 90% (*β* 10%), using as a reference the study of Sheng et al. [13].

The Human Ethics Committee of the *Universidade Federal de Santa Maria* approved this study, and informed consent was obtained from all participants (protocol n. 0169.0.243.000-07).

### 2.2. Materials

Each tablet of Unha de Gato Herbarium contained 100 mg dry *Ut* extract. Biological materials used in the tablets were derived from plants in their natural habitat. The *Ut* extract was prepared by ultra-turrax extraction (Biotron, Kinematica AG) from ground bark (Centroflora) using 70% ethanol (Dipalcool). The HPLC analysis of *Ut *dry extract presents the content of 2.57% pentacyclic oxindole alkaloids (POAs), which were calculated with reference to external calibration curves of mitraphylline. The analysis of extract showed absence of tetracyclic oxindole alkaloids in the sample, allowing its use for therapeutic and research purposes in accordance with U.S. Pharmacopeia.

### 2.3. Sample Collection

Blood was collected in citrated, EDTA, heparin, and without anticoagulant Vacutainer tubes, before chemotherapy and after each of the 6 cycles. CAT and SOD activities were determined using whole blood diluted in a 1 : 20 saline solution.

### 2.4. Biochemical Parameters

A COBAS INTEGRA system was used for the quantitative determination of the chemical constituents of the blood, and data were acquired using a COBAS INTEGRA 400 plus apparatus (USA).

### 2.5. Carbonylation of Serum Protein

The carbonylation of serum proteins was determined through a modification of the Levine method [16].

### 2.6. Determination of Lipid Peroxidation

Lipid peroxidation was estimated by measuring TBARS in plasma samples according to a modification of the method of Jentzsch et al. [17].

### 2.7. Catalase (CAT) and Superoxide Dismutase (SOD) Activities

The determination of CAT activity level was carried out in accordance with a modification of the method of Nelson and Kiesow [18]. SOD activity was calculated based on the ability to inhibit the reaction of superoxide and adrenaline, as described by McCord and Fridovich [19].

### 2.8. Hemograms

Blood samples were analyzed using a Pentra apparatus (France). The lowest values were confirmed by observation of slides using May Grünwald-Giemsa stain and optical microscopy.

### 2.9. Interleukin 6 (IL-6)

ELISA assays of IL-6 were carried out according to a previously published method [20] at room temperature in 96-well microtitre plates (Nunc-Immuno Plate Maxi Sorp), and optical densities (O.D.) at 490 nm were determined using a microplate reader (Thermo Scientific Multiskan FC, Vantaa, Finland).

### 2.10. Single Cell Gel Electrophoresis (Comet Assay)

Alkaline comet assays were performed as described by Singh et al. [21]. One hundred cells (50 cells from each of the two replicate slides) were selected and analyzed. The slides were analyzed under blind conditions by at least two different individuals.

### 2.11. CD3^+^, CD4^+^, and CD8^+^ Cells

Samples were collected in EDTA, and analyses were performed using a three-color fluorescence-activated cell sorter (FACScalibur, Becton Dickinson Biosciences, USA) and Multiset software (Becton Dickinson). FITC-conjugated anti-CD4, PE conjugated anti-CD8 and PerCp conjugated anti-CD3 were used. Immune subpopulations were measured as a percentage of the total number of CD3^+^ cells.

### 2.12. Adverse Events

The Common Terminology Criteria for Adverse Events (AE) v3.0 (CTCAE) from the National Institutes of Health/National Cancer Institute-EUA [22] has been used. Grade refers to the severity of the AE. The CTCAE v3.0 employs grades from 1 to 5, with unique clinical descriptions of severity for each AE based on the following general guideline: grade 1, mild AE, grade 2, moderate AE, grade 3, severe AE, grade 4, life-threatening or disabling AE, and grade 5, death related to an AE. The adverse events were judged in terms of clinical symptoms by interview at each chemotherapy cycle with pharmaceutical. Serum clinical chemistry, whole blood analysis, and leukocyte differential counts were also used to monitor the efficacy and toxicity by physicians of the Department of Oncology.

### 2.13. Statistics

Data were analyzed using the EpiInfo computer program, version 3.5.1 from the CDC, USA. The data were evaluated using analysis of variance (ANOVA) and *t*-test and were expressed as a mean ± SD. When the variances were not homogenous and ANOVA was not appropriate (Bartlett's *P* value < 0.05), Wilcoxon two-sample test was used to evaluate the data. *P* < 0.05 was considered statistically significant.

## 3. Results

The general characteristics of colorectal cancer patients included in this study are shown in Table 1. The mean age of the C group was 60.89 years, and the mean age of the UT group was 62.68 years old.

One aim of the study was to evaluate the neutropenia, thrombocytopenia, and anemia. The hemograms were analyzed each 15 days, and there were no significant differences in hematological parameters (Tables 2 and 3) between the groups for any of the cycles examined. An important reduction in white blood cells (WBCs) count was observed in both groups along the treatment. Unlike what was observed in leukocytes, red blood cells (RBCs) showed recovery of the hypochromic and microcytosis present at baseline. Erythrocyte indices (mean corpuscular hemoglobin-MCH; mean corpuscular volume, MCV) improved in both groups, reaching normal values.

The generation of ROS may damage all types of biological molecules. Oxidative damages to lipids, proteins, or DNA were evaluated by TBARS levels, protein carbonyl levels, and comet assay, respectively. Antioxidant defense system was measured by activity of antioxidants enzymes catalase and SOD. The *Ut* supplementation did not change oxidative stress values or activity of the antioxidant enzymes. Similarly, the comet assay, a sensitive technique for the detection of DNA damage at the level of the individual eukaryotic cell, demonstrated no differences between groups (Table 4).

The CD4^+^ T cells and CD8^+^ T cells (absolute count and ratio) used for the evaluation of the immune status of CRC patients were not statistically different following *Ut* supplementation (Table 5) or chemotherapy (before treatment began versus after the sixth FOLFOX4 cycle). The UT and C groups showed differences before chemotherapy in IL-6 levels, but such differences did not change over the course of treatment. Moreover, in the comet assays, IL-6 levels showed large variations between subjects.

The assessment of adverse events (AEs) related to treatment was conducted by interviewing the patients during each cycle of chemotherapy and through analysis of laboratory tests and observation of abnormal symptoms presented by patients. AEs were classified according to the Common Terminology Criteria for Adverse Events v3.0 (CTCAE v3.0) [22]. Since there were no differences between groups, data shows that *Ut* supplementation did not alter the occurrence of AEs, related to chemotherapy, neither caused AE. The most frequently observed AE in both groups were fatigue, nausea, and a decrease in hematological parameters (Tables 6 and 7). An important reduction in neutrophils (grade 3 or 4) occurred in 25.4% of patients. Toxicity of the *Ut* was also evaluated using liver, kidney, metabolic, and constitutive parameters. Treatment with *Ut* did not alter liver function, defined as elevation of liver enzymes (alanine aminotransferase-ALT, aspartate aminotransferase-AST, *γ* glutamyl transpeptidase-GGT), and bilirubin levels, and kidney function is evaluated by dosage of urea, metabolic parameters (albumin levels and glycemia), and constitutive parameters (weight loss) (data not shown). There was a small difference in creatinine levels between groups before treatment (UT = 74.25 *μ*mol/L, C = 68.95 *μ*mol/L), which remained at the sixth cycle of treatment (UT = 76.90 *μ*mol/L, C = 60.12 *μ*mol/L).

## 4. Discussion

Complementary and alternative medicine (CAM) has been used by a large number of cancer patients worldwide. Cultural, socioeconomic, and spiritual differences affect the rate of use. For instance, there are high rates of use in Mexico (97.2%) and China (97%) [23, 24], an intermediate rate of use in the USA (63%) [25], and lower rates of use in Canada (47%) [26] and Iran (35%) [27]. The herbal remedy cat's claw is used as CAM by some cancer patients. It is thought to be an anticarcinogen, an immunostimulant, and an antioxidant that can stimulate DNA repair. Despite a theoretical understanding of its mechanism of action, the evidence for its clinical effectiveness is minimal [28].

To evaluate the effectiveness of *Ut* in minimizing the main side effects of chemotherapy, a decrease in neutrophil and platelet counts, hemograms were analyzed before each FOLFOX4 cycle (at an interval of 15 days). Treatment with *Ut* was suspended on the days that patients received chemotherapy, because some antineoplastic drugs and CAMs are metabolized through the cytochrome P450 family, and an interaction could alter the metabolism of patients [28]. Treatment with *Ut* did not improve the WBC, RBC, or platelet counts, because there were no differences between groups (UT versus C). *In vivo* assays in rats undergoing chemotherapy demonstrated that neutrophils recover significantly sooner with *Ut* supplementation [14]. This effect of *Ut* on WBC is due both to the stimulation of myeloid precursors [12] and the effect on ROS, which increases survival of lymphocytes [29] and inhibits myeloid cell differentiation [2]. We did not find other clinical trials with CRC patients using *Ut*. In a human volunteer study, *Ut* extract was given at 250 or 350 mg/day for 8 consecutive weeks to healthy adult. There were no statistically significant differences among the groups in WBC [11]. Our group conducted a clinical trial of women with breast cancer undergoing chemotherapy treatment who received 300 mg of *Ut* daily. In this study, we found significant differences between the group that received *Ut *and the control group; the *Ut* group showed higher neutrophils counts compared with the control group (unpublished data). The differences in the drugs used in the treatment of breast cancer (5-FU, adriamycin, and cyclophosphamide) versus CRC (5-FU and oxaliplatin) have to be considered, as do the differences in time between cycles of chemotherapy (21 versus 15 days). We must also consider the fact that all CRC patients in the present study underwent colectomy, which could interfere with the absorption of *Ut*.

Many previous studies have clearly shown the potential of the antioxidant *Ut*, and its potent radical scavenger activity was confirmed by several assays including the following: the capacity to reduce the free radical diphenylpycrilhydrazyl (DPPH assay) [30, 31], the reaction with the superoxide anion, peroxyl [30], and hydroxyl radicals [30] as well as with the oxidant species, hydrogen peroxide, and hypochlorous acid [30, 32], and the TEAC assay [10]. The antioxidant activity of *Ut *extracts was further assayed through determination of TBARS production (using rat liver homogenates and sarcoplasmic reticulum membranes) and by the inhibition of free radical-mediated DNA-sugar damage [30, 33]. These assays were primarily *in vitro* tests with one *in vivo* test [31]. Despite this strong evidence, no differences in oxidative stress were found between groups that received or did not receive *Ut*, as assessed by lipid peroxidation (TBARS) and protein carbonyls. In addition, no differences were observed in the antioxidant enzymes SOD or catalase. 

There are close correlations between DNA damage, DNA repair, and immune responses in lymphocytes. DNA damage and mutations may result in a failure of T cells to proliferate and undergo extensive clonal expansion upon antigenic stimulation. Sheng et al. [11] showed that a water-soluble extract of *Ut* caused a significant decrease in DNA damage and a concomitant increase in DNA repair in volunteers. However, in our study, the comet assay did not demonstrate a significant difference in the group that received *Ut*. *Ut *extract was prepared through an extraction of ground bark with 70% ethanol. This process altered the composition of the extract (oxindole alkaloids) compared with an aqueous extract (like that used by Sheng et al. [11]). However, more recently, water-soluble cat's claw extract was shown not to contain significant amounts of alkaloids (<0.05%). Yet, it was still shown to be efficacious, because quinic acid is the major active ingredient [34]. Further study is needed to assess whether differences in the content of the extracts are correlated with the differences in observed results. 

Similar to oxidative stress, *Ut* did not show an effect on the analyzed immunologic parameters, the CD4^+^ T cell-CD8^+^ T cell count and the IL-6 levels despite the *in vitro* evidence [35].

There were no drug-related toxic effects observed for *Ut* extract at a repeated dose of 300 mg/day for 12 consecutive weeks (Unha de Gato Herbarium), when judged in terms of clinical symptoms, serum clinical chemistry, whole blood analysis, and leukocyte differential counts. Similar results have been shown in previous studies with volunteers [11, 36]. National Center for Complementary and Alternative Medicine (USA) [37] has reported few side effects from cat's claw at the recommended dosages. Though rare, side effects may include headaches, dizziness, and vomiting.

Adverse events related to antineoplastic drugs (oxaliplatin and 5FU) are well known [1] and are similar to those observed in our study.

## 5. Conclusion

*Ut *at dose 300 mg dry extract daily is not effective in reducing the most prevalent adverse events due to treatment with 5FU/Leucovorin and oxaliplatin in patients with advanced CRC. No toxic effects related to *Ut* were observed in the group that received 300 mg dry extract daily for 12 weeks. Additional studies are needed to evaluate under which conditions, drugs, or types of cancer *Ut* might have a positive effect on treatment, in decreasing neutropenia and thrombocytopenia, or in improving the immune response.

##  Conflict of Interests

All the authors deny any conflict of interests. This work had a financial support from the government agencies CNPq and CAPES.

## Figures and Tables

**Table 1:** General data of the CRC patients in adjuvant/palliative chemotherapy (FOLFOX4) without *Uncaria tomentosa *supply (C group) or receiving 300 mg/day of *Uncaria tomentosa* (UT group).

*Parameters*		*C group* *n* = 23	*UT group* *n* = 20
^ a^States T	T1	0	1
	T2	1	1
	T3	16	12
	T4	6	6

^ a^States N	N0	1	2
	N1	8	8
	N2	11	10

^ a^States M	M0	13	17
	M1	10	3

Age	<50	4	2
	51–65	10	12
	66–80	9	6

Gender	Female	16	10
	Male	7	10

Smoke	Smokers	2	0
	ex-smokers	8	10
	no smokers	13	10

Associated chronic diseases	Without	5	4
	Hypertension	6	6
	Hypertension + coronary diseases/dyslipidemia/diabetes	3	7
	Diabetes	2	2
	Others	4	1

^a^Stage of disease currently described by TNM, as published by the American Joint Committee on Cancer (AJCC) and American Cancer Society (ACS).

**Table 2:** Evaluation of hemoglobin, and erythrocyte indices of the CRC patients, during six cycles of adjuvant/palliative chemotherapy, without *Uncaria tomentosa *supply (C group) or receiving 300 mg/day of *Uncaria tomentosa* (UT group).

*Parameters*	*Group*	*Chemotherapy cycle*						
		0	1	2	3	4	5	6
Hb	UT	123.5	125.2	127.2	123.5	125.3	121.4	118.6
g/L		(14.9)	(17.9)	(17.0)	(14.2)	(13.9)	(11.1)	(10.4)
	C	113.7	115.1	113.3	113.9	114.9	117.0	113.7
		(17.6)	(13.8)	(15.7)	(17.2)	(14.2)	(12.5)	(14.2)
MCH	UT	27.53	27.88	28.37	28.95	29.66	29.69	30.60*
pg		(1.99)	(1.69)	(1.97)	(2.20)	(2.31)	(1.92)	(2.16)
	C	26.62	27.02	27.37	27.70	27.93	28.80	29.19*
		(2.61)	(2.63)	(2.59)	(2.67)	(2.63)	(2.60)	(2.44)
MCV	UT	84.62	85.31	86.03	87.57	89.13	90.00	91.50**
fL		(4.31)	(3.91)	(3.65)	(5.36)	(5.59)	(4.90)	(4.84)
	C	81.94	82.53	83.74	85.28	86.27	88.29	89.22**
		(6.8)	(6.58)	(6.4)	(6.34)	(6.02)	(5.92)	(5.51)

Values expressed as mean (SD). Hb: hemoglobin, MCH: mean corpuscular hemoglobin, MCV: mean corpuscular volume. UT group: patients treated with FOLFOX4 + *Uncaria tomentosa* 300 mg/day (*n* = 20), C group: patients treated with FOLFOX4 (*n* = 23); *P < 0.05; **P < 0.001; ***P < 0.0001 in relation to the day 0.

**Table 3:** White blood cells count and platelets's evaluation of the CRC patients in adjuvant/palliative chemotherapy, without *Uncaria tomentosa *supply (C group) or receiving 300 mg/day of *Uncaria tomentosa* (UT group).

*Parameters*	*Groups*	*Chemotherapy cycles*						
		0	1	2	3	4	5	6
WBC	UT	8.178	5.689*	5.184**	4.778**	4.956**	4.660**	4.442**
cells ×10^9^/L		(2.705)	(1.919)	(2.051)	(2.022)	(2.006)	(2.095)	(2.433)
	C	7.668	5.933*	5.391*	4.886*	4.473***	4.962**	4.195***
		(2.892)	(2.137)	(2.451)	(2.039)	(2.086)	(2.157)	(1.558)
Neutrophils	UT	5.345	3.069*	2.600**	2.441**	2.429**	2.227**	2.343***
cells ×10^9^/L		(2.691)	(1.455)	(1.411)	(1.401)	(1.456)	(1.506)	(1.842)
	C	4.871	3.285*	2.848**	2.295***	2.190***	2.514*	1.975***
		(2.674)	(1.618)	(1.858)	(2.295)	(1.628)	(1.797)	(1.186)
Lymphocytes	UT	2.038	1.888	1.859	1.673	1.776	1.728	1.433*
cells ×10^9^/L		(.735)	(.681)	(.656)	(.642)	(.661)	(.754)	(.504)
	C	1.901	1.888	1.815	1.769	1.650	1.697	1.578
		(.702)	(.737)	(.717)	(.827)	(.648)	(.531)	(.659)
Monocytes	UT	.538	.515	.528	.482	.546	.547	.542
cells ×10^9^/L		(.215)	(.157)	(.197)	(.216)	(.244)	(.241)	(.306)
	C	.542	.533	.570	.602	.470	.595	.498
		(.245)	(.254)	(.254)	(.272)	(.197)	(.262)	(.231)
Platelets	UT	263	188*	174*	146***	135***	117***	117***
count ×10^9^/L		(92)	(43)	(55)	(48)	(51)	(42 )	(33)
	C	286	216*	197**	161***	149***	165***	141***
		(76)	(68)	(64)	(70 )	(66)	(57)	(58)

Values expressed as mean (SD). UT group: patients treated with FOLFOX4 + *Uncaria tomentosa* 300 mg/daily (*n* = 20); C group: CRC patients received FOLFOX4 (*n* = 23); *P < 0.05; **P < 0.001; ***P < 0.0001 in relation to the day 0.

**Table 4:** Evaluation of lipid peroxidation, carbonylation of serum protein, DNA damage and antioxidant defenses of the CRC patients in adjuvant/palliative chemotherapy (FOLFOX4), without *Uncaria tomentosa *supply (C group) or receiving 300 mg/day of *Uncaria tomentosa* (UT group).

*Parameters*	*Group*	*Chemotherapy cycles*						
		0	1	2	3	4	5	6
TBARS nmol	UT	16.7	16.2	18.3	17.9	17.7	17.8	21.6
MDA/mL		(9.34)	(7.1)	(7.2)	(6.9)	(4.1)	(3.4)	(11.8)
	C	22.5	18.8	17.8	19.4	21.2	22.4	22.9
		(11.6)	(10.9)	(11.3)	(10.5)	(8.9)	(9.7)	(10.5)
Protein carbonyl	UT	0.63	0.56	0.61	0.61	0.68	0.67	0.6
nmol/mg protein		(0.2)	(0.2)	(0.17)	(0.18)	(0.26)	(0.2)	(0.2)
	C	0.79	0.77	0.73	0.72	0.78	0.9	0.84
		(0.37)	(0.4)	(0.39)	(0.36)	(0.37)	(0.43)	(0.37)
Comet assay	UT	29.04						26.78
Index damage		(34.18)						(31.99)
	C	26.94						34.66
		(49.3)						(46.63)
Catalase	UT	7.85	8.2	7.65	9.12	8.97	9.33	10.39
pmol/mg protein		(3.3)	(3.0)	(2.81)	(4.75)	(4.71)	(3.27)	(4.08)
	C	9.05	8.29	8.51	8.06	9.07	8.31	9.38
		(4.9)	(2.7)	(4.05)	(3.51)	(3.71)	(3.07)	(3.78)
SOD	UT	1.82	1.85	1.95	2.19	1.95	2.29*	2.41*
U/mg protein		(0.5)	(0.44)	(0.44)	(0.43)	(0.43)	(0.44)	(0.56)
	C	1.91	1.91	2.1	2.15	2.09	2.12	2.13
		(0.8)	(0.76)	(0.71)	(0.78)	(0.7)	(0.81)	(0.72)

Data expressed in mean (SD). TBARS, thiobarbituric acid-reactive substances; SOD, superoxide dismutase; UT group: patients treated with FOLFOX4 + *Uncaria tomentosa* 300 mg/daily (*n* = 20); C group: CRC patients received FOLFOX4 (*n* = 23). *P < 0.05 in relation to the day 0.

**Table 5:** Immune status of CRC patients before treatment began and after 6 cycles of adjuvant/palliative chemotherapy (FOLFOX4) without *Uncaria tomentosa *supply (C group) or receiving 300 mg/day of *Uncaria tomentosa* (UT group).

*Parameters*	*Group*	*Chemotherapy cycles*	
		0	6
CD4^+^ T Cells	UT	958.36 (414.6)	720.28 (271.72)
Cells/*μ*L	C	828.45 (431.25)	848.38 (430.56)
			
CD8^+^ T cells	UT	494.0 (231.28)	390.64 (223.62)
Cells/*μ*L	C	490.29 (271.14)	394.27 (149.96)
CD4^+^ T/CD8^+^ T Ratio	UT	2.17 (0.76)	2.21 (0.78)
	C	1.96 (1.03)	2.30 (1.08)
IL6	UT	4.07^#^ (6.54)	5.1^#^ (6.12)
ng/mL	C	12.97 (13.28)	16.66 (18.2)

Data expressed as mean (SD); UT group: patients treated with FOLFOX4 + *Uncaria tomentosa* 300 mg/daily (*n* = 20); C group: CRC patients received FOLFOX4 (*n* = 23). ^#^ *P* < 0.05 between groups.

**Table 6:** Frequency of side effects reported by CRC patients in adjuvant/palliative chemotherapy in interview at first and sixth cycle of the treatment.

	*After 1 chemotherapy cycle*					*After 6 chemotherapy cycles*				
	Not present	rarely	sometimes	often	Always	Not present	Rarely	Sometimes	Often	always
Fatigue	60.5	13.2	13.2	5.3	7.9	54.3	5.7	22.9	5.7	11.4
Insomnia	86.8	2.6	7.9	2.6	0	97.1	2.9	0	0	0
Vomiting	78.9	10.5	10.5	0	0	100	0	0	0	0
nausea	60.5	15.8	21.1	2.6	0	80.0	15.0	0	0	5.0
Dry skin	91.2	2.9	2.9	2.9	0	88.6	0	0	5.7	5.7
Pruritus/itching	81.6	2.6	10.5	0	5.3	91.4	5.7	0	0	2.9
Fever	97.4	2.6	0	0	0	97.1	2.9	0	0	0

Data expressed as % of the patients who had symptoms.

**Table 7:** Adverse events observed in CRC patients in adjuvant/palliative chemotherapy with FOLFOX4 (*n* = 43).

	*After 1 chemotherapy cycle (FOLFOX4)*					*After 6 chemotherapy cycles (FOLFOX4)*				
	Grade refers to the severity of the AE*					Grade refers to the severity of the AE				
	0	1	2	3	4	0	1	2	3	4
Hemoglobin	82.9	12.2	4.9	0	0	76.9	17.9	2.6	0	0
Leukocytes (total WBC)	97.6	2.4	0	0	0	74.4	5.1	15.4	5.1	0
Neutrophils/granulocytes	85.4	7.3	0	4.9	2.4	48.7	12.8	10.3	17.9	7.7
Lymphocytes	95.1	0	4.9	0	0	92.3	0	7.7	0	0
Platelets	97.6	0	2.4	0	0	84.6	10.3	5.1	0	0
Weight loss	82.9	9.8	2.4	4.9	0	92.3	0	2.6	5.1	0
Hyperglycemia	97.6	0	0	2.4	0	87.2	0	7.7	5.1	0
*γ*-glutamyl transpeptidase	100	0	0	0	0	89.8	10.2	0	0	0
Alkaline phosphatase	100	0	0	0	0	84.6	15.4	0	0	0
Neuropathy: sensory	100	0	0	0	0	94,9	0	5.1	0	0
Infection with Grade 3 or 4 neutrophils	100	0	0	0	0	97.4	0	2.6	0	0
Diarrhea	100	x	0	0	0	92.3	x	7.7	0	0

Values expressed as % of the patients who had AE. *Grade refers to the severity of the AE: grade 1 = mild AE; grade 2 = moderate AE; grade 3 = severe AE; grade 4 = life-threatening or disabling AE; grade 5 = death related to an AE [22].
